# Radiation Exposure of Crystalline Bodies during Interventional Therapy and Related Research Status

This article has been retracted.

**DOI:** 10.1155/2022/5480409

**Published:** 2022-07-31

**Authors:** Yahong Chen, Dong Zhao, Hongwei Zhong, Yiheng Zhang, Donghong An

**Affiliations:** ^1^Catheter Room, China-Japan Union Hospital of Jilin University, Changchun, Jilin 130031, China; ^2^Department of Radiological Intervention, China-Japan Union Hospital of Jilin University, Changchun, Jilin 130031, China

## Abstract

The aim of this study was to estimate the exposure dose level of ocular corpuscles during the common interventional procedures of interventional radiology workers. This article retrospectively analyzed the general instruments and equipment of interventional therapy, the general methods and steps of interventional therapy, and the influence of X-ray of interventional surgery. The related contents of eye protection for interventional radiology workers were summarized. This study found that there was a significant linear correlation between the equivalent dose of lens and the exposure time. The tube voltage, tube current, and the size of fluoroscopic field of vision also have an impact on the radiation of workers during surgical exposure. Interventional surgery is difficult and easy. The exposure time of difficult surgery is relatively long, so the dose received by interventional staff is large. The intervention staff should improve their professional knowledge, be proficient in the operation technology, and try to reduce the exposure without affecting the diagnosis and treatment effect. During the intervention operation, the eye substance of the operator is exposed to a certain dose of radiation, and the wearing rate of protective lead glasses of the intervention staff is very low. Therefore, we must pay attention to the protection of the eyes, strengthen the protection management, and reduce the exposure dose of the intervention staff as much as possible.

## 1. Introduction

With the continuous progress of medical technology, interventional therapy is becoming more and more common, and there are more and more interventional operations, so radiation protection has become a key work [1]. Through the publicity and training of radiation protection in recent years, the self-protection awareness of the involved staff has been strengthened, including the use of lead clothes, lead neck covers, lead hats, and lead glasses. In various organs and tissues of the body, the eye lens is one of the tissues sensitive to radiation. Long-term exposure to low-dose ionizing radiation will damage the lens capsule, and water will enter the lens, which can cause eye lens turbidity and even lead to radioactive cataract, seriously affecting life. The use of lead protective glasses can greatly reduce the damage to eyes caused by radiation. In fact, eye protection is a weak link in radiation protection. A large number of interventional workers do not wear lead protective glasses during surgery, resulting in direct exposure of eyes to radiation. In order to make interventional radiology workers aware of the harm of radiation to eye lens, enhance their awareness of eye protection at work, reduce radiation dose, and ensure their health [2].  Figure 1 shows percutaneous coronary intervention. Interventional surgery can be divided into intravascular intervention and nonintravascular intervention. Intravascular intervention refers to the use of a puncture needle to reach the human vascular system through the superficial arteries and veins of the human body. Under the guidance of the angiography machine, the surgeon will send the catheter to the desired position according to his own knowledge of human anatomy. Under the development of the angiography agent, the vascular condition of the lesion can be determined, and the lesion can be treated directly in the blood vessel [3], including arterial embolization and angioplasty. Commonly used body surface puncture points include radial artery, femoral artery, femoral vein, subclavian artery, subclavian vein, carotid artery, and vein. Nonvascular intervention refers to the method that the puncture needle and catheter do not directly enter the vascular system, but puncture the lesion through the skin or directly enter the lesion through the normal channel of the human body with the help of relevant imaging equipment, so as to treat the lesion, including intratumoral drug injection, percutaneous tumor biopsy, intervertebral disc puncture ablation, and intervertebral disc puncture decompression.

## 2. Literature Review

Aiming at this research problem, Opitz and others used TDL to compare the radiation dose of eye lens in the two chest photography positions of prone posterior-anterior position and supine anterior-posterior position and to explore whether there is any difference in the radiation dose of eye lens in the two chest photography positions [4]. Mantis and others believe that the mechanism leading to no coronary reflow during PCI is mainly related to microvascular circulatory dysfunction. Endothelial dysfunction, endothelial glycocalyx injury, inflammatory reaction and oxidative stress, platelet activation, mechanical obstruction caused by leukocytes or immune cells, hypercholesterolemia, excessive dose of contrast agent, etc., are related factors that lead to no reflow of coronary artery during PCI, while thrombus aspiration and IABP may be the related factors that reduce no reflow of coronary artery during PCI [5]. Boeri and others investigated the current situation of the sense of personal control of young and middle-aged patients after PCI and analyzed its influencing factors, in order to provide reference for the psychological rehabilitation intervention of young and middle-aged patients after PCI [6]. Riaz and others investigated the current situation of health literacy of patients after the first PCI and analyzed its influencing factors, in order to provide reference for the formulation of health literacy intervention strategies for patients after the first PCI [7]. Pop and others investigated the workers engaged in ionizing radiation and 840 workers engaged in nonionizing radiation. Through the analysis of lens changes, they can judge whether they are affected by ionizing radiation and provide a basis for clinical prevention of ionizing radiation. The method shown in Figure 2 exists in radiation [8]. Kong and others believe that after the human body is affected by radiation, gender, central nervous system, and long-term exposure to radiation, it can lead to cataract. Therefore, it is very important to detect lens damage for personnel engaged in ionizing radiation. However, the inference results of high-dose and medium-dose radiation cannot accurately reflect the real situation of low-dose radiation. Therefore, it is necessary to understand the impact of low-dose ionizing radiation on the lens of relevant workers, so as to provide the most direct basis for detecting the health risk data of ionizing radiation related people [9].

Based on the current research, this paper aims to estimate the exposure dose level of ocular corpuscles in the common interventional procedures of interventional radiology workers. This paper retrospectively analyzed the general instruments and equipment of interventional therapy, the general methods and steps of interventional therapy, and the influence of X-ray of interventional surgery. The related contents of eye protection for interventional radiology workers were summarized. The retrospective analysis showed that there was a linear correlation between the equivalent dose of lens and the length of exposure time; interventional surgery is difficult and easy. The exposure time of difficult surgery is relatively long, so the dose received by interventional staff is large. The intervention staff should improve their professional knowledge, be proficient in the operation technology, and try to reduce the exposure without affecting the diagnosis and treatment effect.

## 3. Analysis

### 3.1. General Instruments and Equipment for Analysis of Interventional Therapy

Thermoluminescence dosimeter used in this investigation is a special thermoluminescence dosimeter for eye lens. The eye body dosimeter is equipped with two kinds of ring covers, which can directly place the detector in the plastic tank equivalent to the tissue for monitoring. The color of the dosimeter is green. When reading after monitoring, the detector can be taken out of the plastic tank. In the experimental monitoring, only one piece of thermoluminescence detector is used in each eye body dosimeter. The dosimeter is small in size and light in weight. When the interventional physician wears it for operation, there will be no discomfort, so as to avoid adverse effects on the operation due to discomfort. Therefore, the thermoluminescence dosimeter has the characteristics of simple operation, moisture-proof, and waterproof without affecting the operation and monitoring results. GR-200 A thermoluminescence detector is LIF (Mg, Cu, P) sheet type. The diameter of the detector is 3.6 mm, the thickness is 0.4 mm, and the dispersity is <2.0%.

Interventional equipment: Philips allura 12&15 digital subtraction angiography machine, German Siemens aritiszee angiography machine and Philips large flat plate angiography machine FD20. The three interventional equipment are under bed ball tubes, and the tube current and tube voltage can be automatically adjusted and are equipped with movable hanging lead protective curtain.

### 3.2. Analyze the General Methods and Steps of Interventional Therapy

1. Preparation of thermoluminescence dosimeters: the thermoluminescence dosimeter (tablet type) is placed in a glass dish, annealed in a 2000b TLD far infrared precision annealing furnace at 240°C for 10 min, and taken out and cooled naturally. The thermoluminescence dosimeter is placed in the dosimeter wearing clip for use.
2. Methods before operation: the dosimeter clip prepared in advance was worn near the left eye of the surgical cap of the first and second operators. Relevant data were recorded during the operation, such as operation date, name, tube voltage, tube current, operation exposure time, and air specific release kinetic energy. After each operation, remove the dosimeter clip, place it in different fresh-keeping bags, mark it, take it back to the laboratory, measure it with rgd-3b thermoluminescence meter, and record the data.

### 3.3. Impact of X-Ray in Interventional Surgery

As we all know, interventional surgery has become a very important way of diagnosis and treatment, which is indispensable in clinical practice. The interventional therapy technology in China started relatively late. However, due to the large population, the interventional surgery has developed rapidly and the technology has been continuously improved. In recent years, the number of intracardiac interventional surgery in China has maintained an average annual growth rate of 20%–30%. With the gradual popularization of interventional surgery, the number of staff engaged in interventional work is also increasing. The interventional staff will inevitably be exposed to X-ray irradiation during the interventional operation. Due to long-term exposure to low-dose X-ray irradiation, the radiation will produce a series of damage effects on the body and have a harmful impact on the health of the staff exposed to X-ray. As interventional workers have more knowledge about radiation effects and radiation protection, the radiation protection of interventional surgeons has further attracted the attention of the general public and relevant departments [10, 11]. The use of various radiation protection facilities, such as the use of movable lead protective hanging curtains, lead clothes, lead bibs, and lead protective glasses, has greatly reduced the exposure dose of intervention workers to a certain extent, and ensured the health of intervention workers [12]. In the above-mentioned radiation protection measures, most of the protective facilities are in place and have achieved good protection effects [13, 14]. However, the use rate of lead protective glasses is very low. It has been reported that the use rate of lead protective glasses for interventional surgeons is less than 70%.

X-ray is widely used in the medical field, almost involving all aspects of medical treatment. In the medical field of X-ray application, X-ray related workers are more or less inevitably exposed to X-ray radiation and have certain adverse effects on their own health. In clinical practice, interventional doctors are radiation workers who are more exposed to X-rays. The nurses in the catheter room will only assist in the operation on the operating table in individual cases of individual operations. Therefore, the dose received is very small [15].

In the retrospective analysis and investigation of eye lens dose, the dosimeter was worn in front of the subject's chest or neck, which was far away from the eyes, and the monitoring results were inaccurate. In this retrospective analysis, the thermoluminescence dosimeter was placed near the left eye of the surgical cap, which was very close to the eye. Therefore, the data obtained were relatively accurate [16, 17]. In the process of surgical exposure, the intervention staff will receive a certain dose of radiation, especially the coronary angiography + stent implantation in the cardiac intervention. Stent implantation is originally a difficult operation. The general shape of the coronary artery is fixed, but individual cases also vary from person to person. In addition, the severity of the patients' diseased vessels varies, and the operating skill of the surgeons varies. Therefore, due to many uncertain factors in the process of stent implantation, the dose rate and total exposure time of radiation exposure during the operation are different, and the dose received by the eye lens of the operator is also different [18]. Intervention workers are directly exposed to radiation at work. If there is no protective effect of relevant protective facilities, it is easy to exceed the dose threshold specified in relevant documents, and it is very likely to cause irreversible radiation damage and seriously affect their health [19, 20].

### 3.4. Eye Protection of Interventional Radiation Workers

With the development of interventional surgery, the protection of interventional workers has been paid more and more attention by the society. The personal protection of interventional radiology workers is the premise and primary principle to ensure the safe and smooth development of interventional diagnosis and treatment and continue to benefit patients [21]. Only when the health of the intervention staff is guaranteed, can they devote themselves to their work and provide the best service for patients. Eye protection for intervention workers has always been a weak link in protection. Therefore, eye protection should be the key work in current protection [22].

In interventional surgery, the vast majority of interventional surgery workers' eyes are directly exposed to radiation, and there are many reasons why they do not wear lead protective glasses. However, in the final analysis, their awareness of eye protection is too poor, and they have an indifferent or irrelevant attitude [23, 24]. Although they have all received prejob radiation protection related training and learned about the impact of radiation on the body, the protection of eyes is not in place. Therefore, in the next step, the first thing to do is to strengthen the protection awareness of intervention workers, especially the eye protection awareness, and then fundamentally emphasize the importance of their own eye protection, so as to solve the dilution of eye protection awareness and strive to greatly improve the wearing rate of protective glasses [25].

### 3.5. Relevant Departments of the Hospital Shall Strengthen Management

Lead protective glasses are the last protective barrier for eye protection and are indispensable. In this investigation, a large number of people do not have lead protective glasses, partly because they are expensive. Therefore, in order to do a good job in the protection of intervention workers, the relevant departments of the hospital should do a good job in publicity and supervision. At the same time, the management of the radiology department of each hospital should establish a complete physical examination file for the radiology staff and do a good job in the health examination of the radiology staff.

### 3.6. Health Supervision Departments Should Strengthen Supervision

The health supervision and management department shall strengthen the protection supervision and management of radiation workers. For units, departments, or individuals, whose protection is not in place, relevant measures shall be taken, strict requirements shall be imposed, and supervision shall be raised to a higher level to ensure no omission.

### 3.7. Improvement of Lead Protective Glasses

A large part of the intervention personnel have protective glasses, but they almost never wear them. The reason is that the quality of lead protective glasses is too heavy, so it is very inconvenient to wear them. During the operation, the wearing of lead protective glasses can even affect the operator's mood, affect the normal operation of the surgeon, and even seriously affect the operation results. If the surgeon does not wear protective glasses, his health will not be guaranteed while he treats the patient. In the long run, his eyes are likely to have radioactive cataracts, which will seriously affect his quality of life. Therefore, the interventional doctor must wear protective glasses during the interventional operation. If we can design lightweight protective glasses, or they are not different from ordinary glasses, it will be a blessing for interventional doctors. However, the current level of science and technology is very limited, and it is not possible to design and manufacture ideal protective glasses or eye protection facilities. Therefore, the research and development of lead protective glasses is imperative.

### 3.8. Use of Lead Protective Hanging Curtain

This investigation found that the equivalent dose of lens of the interventional workers who were close to the bulb tube was less than that of the second operator who was far away from the bulb tube. Its main purpose is to use the movable lead protective hanging curtain, which effectively blocks part of the radiation and plays a very good protective role. However, because X-rays have the characteristics of diffraction, surgeons who are shielded by protective hanging curtains will receive part of the radiation. Therefore, the protective hanging curtain still has some shortcomings.

This study found that there was a significant linear correlation between the equivalent dose of lens and the exposure time. The tube voltage, tube current, and the size of fluoroscopic field of vision also have an impact on the radiation of workers during surgical exposure. Interventional surgery is difficult and easy. The exposure time of difficult surgery is relatively long, so the dose received by interventional staff is large. The intervention staff should improve their professional knowledge, be proficient in the operation technology, and try to reduce the exposure without affecting the diagnosis and treatment effect.

## 4. Conclusion

This retrospective analysis found that among several common types of interventional surgery, the equivalent dose received by the interventional workers in the Department of Cardiology was relatively large; in interventional surgery, the equivalent dose of lens in the second operation is often higher than that in the first operation; in the course of interventional surgery, there is a linear correlation between the intraocular lens equivalent dose and the length of surgical exposure; most of the interventional radiology workers do not wear lead protective glasses when working. With the popularization of interventional diagnosis and treatment technology, the radiation protection work has also been continuously improved. The protection of the eye lens of interventional workers still needs further efforts and improvement.

## Figures and Tables

**Figure 1:** Percutaneous coronary intervention.

**Figure 2:** The method of the radiation exists.

## Data Availability

The data used to support the findings of this study are available from the corresponding author upon request.
